RETRACTED

# Evaluation Model of New Socialist Countryside Construction Based on a Multilayer Neural Network in a Complex Environment

**DOI:** 10.1155/2022/9740770

**Published:** 2022-10-08

**Authors:** Guoliang Hou

**Affiliations:** School of Marxism, Weifang University, Weifang 261061, China

## Abstract

The creation of a deep neural network model with numerous hidden layers enables the layer-by-layer extraction of features from the input high-dimensional data, enabling the identification of the data's low-dimensional nested structure and the development of a more efficient and abstract high-level representation. The research on deep learning is thoroughly examined, along with the direction it needs to take going forward. Supporting the construction of new socialist rural areas as a calculated move to address the problems facing farming, rural communities, and farmers is another essential step in furthering modernization. It helps to reshape the entire rural landscape, coordinate the growth of urban and rural areas, achieve the goal of a wealthy society in every way, boost demand, and support the holistic development of people. The emergence of new socialist rural communities against the background of deep learning is the subject of significant research and analysis in this work. In the research, it is examined and studied using deep learning methods and convolutional neural networks. It is evident from the research described in this paper that deep learning backgrounds have a considerable impact on the development of new rural areas—up to 54.53%. In this essay, the foundation for the future construction of a new socialist countryside is laid forth.

## 1. Introduction

Constructing the evaluation index system of building a new socialistic village refers to making an evaluation and judgment on the progress of building a new village by applying certain principles and standards on the basis of comprehensive analysis. It is of great significance to establish a set of evaluation index system with perfect functions, scientific rationality, and simple operation to guide the build of new socialistic village and give full play to the warmth and initiative of the broad masses of the people. Building a new socialistic village is both a practical and a theoretical question. It is necessary to actively explore in practice and systematically study in theory. The present situation is that there are different standards for a new rural area built in different parts of China, which can be described as “each village has its own village standards, each township has its own township standards, each county has its own county standards, and each province has its own provincial standards.” This is bound to make it difficult to assess the effectiveness of new rural build and influence the strength of new socialistic rural build. We should avoid the strange phenomenon that “poor new village” and “rich new village” coexist. The overall goal of promoting the building of new village should be to greatly improve the overall appearance of rural areas and significantly narrow the gap between urban and rural areas in the next 15 years or so [1]. Where does the money come from is a key issue that needs to be resolved in the new rural construction. The central government's investment in “farming, rural areas, and farmers” has expanded more quickly since the proactive fiscal policy's implementation in 1998, accounting for a larger share of the total fiscal spending for supporting agriculture. The total amount of national financial resources available to support agriculture, however, is still insufficient when compared to the demand for new rural construction, and a number of issues, including irrational investment decisions, a subpar management system, an unclear division of investment duties between the central and local public, and the unsatisfactory use of resources, are also significant. In the past, there were limited data in rural areas, and high-resolution remote sensing photos were frequently primarily employed in urban areas with rapid economic expansion. Remote sensing photos may now be interpreted in rural regions thanks to the rapid expansion of remote sensing technology and the significant increase in the data of high-resolution remote sensing photographs. Since the start of the twenty-first century, China has put forth two significant proposals to address issues relating to agriculture, rural communities, and farmers: the first one is to completely abolish the agricultural tax that has existed for more than two thousand years; the second one is to construct a new socialistic village. This signifies the end of the previous era and the start of the next one. It is based on the transition from urban-rural segregation to urban-rural integration [2]. In the study, the deep knowledge algorithm is also studied, and the new rural build of social subject is studied and analyzed based on deep knowledge. Further expanded direction and analysis are made in the domain of deep knowledge. The idea of building a new socialistic village has long appeared. Since the 1950s, this term has often appeared in relevant central important documents and leaders' speeches. New rural build involves economic, political, social, cultural, and other aspects and is a specific rural regional environment. Compared with the traditional rural build, it has certain similarities, but agricultural production is no longer the only way to make a living. The economic sources are increasingly diversified, the industrial build is more sound, the government's attention is obviously enhanced, and the quality of life of rural residents is significantly improved, which fundamentally solves the deep-rooted questions in traditional rural areas [3].

RETRACTED

A significant historical undertaking suggested by the Fifth Plenary Session of the 16th CPC Central Committee is the construction of a new socialist hamlet. It is also a crucial step in closing the gap between urban and rural areas, addressing the issues of farming, rural communities, and farmers, and creating a harmonious community and a society with a moderate level of prosperity. It is crucial to uphold the fundamental tenets of “giving more and taking less,” develop farming through industry, and bring the city to the countryside while creating a new socialist community. Farmers are, nevertheless, the main group involved in creating a new socialist village. The key to increasing the standard of farmers in rural China is to implement a comprehensive plan for creating a society that is moderately prosperous. A recent area of research in machine learning is deep knowledge. Based on neural Internet, a model simulating the analysis and knowledge of human brain is established, which imitates the mechanism of human brain to identify targets and perceive message. The deep knowledge algorithm simulates the thinking process of human brain neurons by CAD and then realizes the function of CAD automatically knowledge data characteristic and completing complex data analysis tasks. In recent years, man-made intelligence products based on deep knowledge algorithm emerge in endlessly, which brings a lot of convenience to our work and life.

In this paper, several study methods are used to study and analyze it. In the study of deep knowledge, the corresponding model diagram and algorithm formula are established to study and analyze it. In the study of socialistic rural build, a number of data maps have been established for further study and analysis. The blaze new trails of this sheet are as follows:

1. In the article, the deep knowledge technology is combined to study and divide the sleeves of the new socialistic village build
2. In the article, the multievidence method is used to study and analyze the build of socialistic village

## 2. Related Work

In order to better promote the build of new socialistic village, we must make clear the difference between the “new village” proposed at present and the previous formulation, understand the connotation and basic characteristics of new socialistic village, make clear the build contents and main tasks, make clear and implement the relationship between scientific expand concept, building a moderately prosperous society in a comprehensive and building a harmonious society, formulate the index system of new socialistic village to clarify the build direction, formulate the measurement standards and monitoring and evaluation methods of new socialistic village, and conduct scientific monitoring and evaluation of the build process to ensure that the new rural build can advance along the normal direction. As a new dimension reduction algorithm of multifloor neural Internet, deep knowledge extracts characteristic from input high-dimensional data floor by floor by building a deep neural Internet model with multiple hidden floors, so as to discover the low-dimensional nested build of data and form a more abstract and effective high-level representation. Starting with the basic principle of deep knowledge algorithm, this paper explains the basic build of single floor Internet of deep knowledge algorithm and its training process in detail. Building a knowledge community in rural areas is a “hematopoietic” innovation project of new rural build, which is of strategic significance for cultivating new farmers who are literate, skilled, and able to operate, improving their overall quality, independent innovation, and self-management ability, and promote the build of community civilization and the expansion of advanced socialistic culture. In order to ensure the needs of promote the build of new socialistic village, it is urgent to give play to the leading role of government investment and establish a diversified investment guarantee mechanism for the build of new socialistic village as soon as possible.

RETRACTED

In the study, Bengio believes that the build of new socialistic village has five major goals, namely, the expansion of rural productivity, the improvement of farmers' living standards, the improvement of rural infrabuild, the expansion of rural social undertakings, and the continued advancement of grassroots democratic politics [4]. Specifically, it is to develop rural productive forces and promote rural economic prosperity; focus on increasing farmers' income and improving farmers' living standards; strengthen the building of democracy and legal system and guarantee the democratic rights of farmers; strengthen the build of spiritual civilization and cultivate new farmers; promote the build of a harmonious society and maintain social stability in rural areas; deepen rural reform in a comprehensive and enhance the vitality of rural expand. Pan et al. think that the main components of building a new socialistic village can be divided into three categories [5]. First, environmental factors are subdivided into financial support for farming, rural infrabuild, rural public utility expansion, rural assistance and social security, urban-rural integration, and coordinated expansion (such as urban-rural economic integration, population integration, social integration, life integration, and ecological environment integration). Second, the basic elements should fully embody the general requirements of “production expand, well-off life, civilized rural style, clean villages and democratic management” and be subdivided into rural economic expand level (or rural productivity level), rural social expand level, rural democratic system build level, and rural spiritual civilization build level. Third, under the effect factors, it is subdivided into farmers' quality level, farmers' material and cultural living standards, farmers' happiness, and so on. The improvement of environmental factors depends on the government's implementation of the policy of “subsidizing farming with industry, bringing villages with cities” and “giving more, taking less, and freeing up the village.” The improvement of basic elements is mainly the question of rural self-build. Sun et al. think that knowledge organization is the new trend of organizational management in the 21st century [6]. The so-called knowledge organization is an organization that innovates itself, improves itself, expands its energy, and responds effectively to the ever-changing external environment across continuous knowledge. Although the community does not have the rigorous build and standard system as an organization, both of them are the social amount to of people who are interrelated and interact with each other in a certain area. Building a rural knowledge community will surely promote the expansion of the community and its members and the build of a new socialistic village. Tang's statement of building a new socialistic village and the guiding ideology of solving the contradiction between urban and rural dual build and coordinating urban and rural expansion proposed by the 16th National Congress of the Communist Party of China for the first time, as well as his repeated statement that solving the “three rural issues” is the top priority of the whole party's work, has always been the fundamental way to curb the widening gap between urban and rural areas, expand rural market demand, and solve the “three rural issues” [7]. Therefore, at present, the content and task of building a new socialistic village are more comprehensive than the previous formulation, which is based on “comprehensively deepening rural reform, stimulating rural vitality, vigorously developing rural productive forces with the support of national policies, speeding up the improvement of rural production and living conditions and overall appearance, and promote rural economic and social expansion.

RETRACTED

## 3. Deep Knowledge Study and Analysis

### 3.1. Study and Analysis of Deep Knowledge Technology

The most popular deep knowledge technologies in the past decade are mostly driven by big data, big calculation, and big model calculation, including Alpha GO and Alpha Zero. Deep knowledge has made great progress in the past period, such as the generated confrontation Internet, transfer knowledge, and GPT-3 proposed in 2020. Its algorithm theory and applied technology need to combine symbolic logic, knowledge reasoning, new paradigm of causality, etc. The deep knowledge algorithm belongs to the category of machine knowledge. Machine knowledge is one of the important branches of man-made intelligence applied. It extracts hidden characteristic of data across algorithms and then realizes data classification and regression, so as to accomplish intelligent identification and prediction. The expansion history of machine knowledge algorithms is divided by different methods according to different people's understanding. With the achievements of deep knowledge in CAD sight, natural speech processing, and other domains becoming more and more remarkable, researchers are discussing it more and more. As far as deep knowledge and man-made intelligence are concerned, most of the innovations in this domain come from large enterprise laboratories of companies such as Google and Microsoft. These companies not only take the lead in impressive study but also regularly open their source codes to simplify the application of man-made intelligence technology. With the continuous expansion and improvement of deep knowledge algorithms, deep knowledge researchers have proposed many mature neural Internet models, which have been widely used in many domains. It is the largest study domain in cognitive science, with more than 10,000 articles on attention phenomenon every year. The attention of the human brain has two important qualities: attention map and dynamic attention mechanism. Among them, there are two kinds of attentional maps: attention salience maps are from bottom-up attentional maps, while attention priority maps combine top-down and bottom-up activities and task relevance. The influence of attention mechanism has also been absorbed by the currently popular directional graph neural Internet, and it has evolved continuously, forming a graph attention Internet architecture. The occlusion self-attention mechanism is used to learn the attention weight between the central node and neighboring nodes, and the spatial message of neighboring nodes is the amount according to the weight to update the feature representation of the central node [8, 9]. Therefore, in the study, a corresponding model diagram is established to analyze and study it, as shown in Figures 1 and 2.

RETRACTED

Deep learning is the process of creating a deep learning model using machine learning. The model is generally accepted to have at least three hidden floors. Because of the large amount of sample data and the slow training process, as well as the fact that the parameters tend to converge on the local rather than the global optimal point, this type of Internet with multiple hidden floors is challenging to train using a common neural Internet, such as the BP algorithm. As a result, the practical significance is weak. Although deep learning and convolutional neural networks are good at extracting and learning data characteristics, when dealing with time-varying data, standard neural network architectures struggle to maintain time series characteristics, which has a number of disadvantages. The time sequence of samples is crucial in applications like natural speech processing and speech admit. Convolution neural Internet, which includes convolution operation floor, pool operation floor, complete connection floor, and admission operation floor, is essentially a multilevel neural Internet, testing the system's knowledge effect with sample data that has never been seen previously by the system, such as the accuracy of sample categorization and the relationship between objective and subjective evaluation. The other floors of deep knowledge, aside from the input and the last floor of output, are concealed, making it difficult to determine how much or what kind of message is held there, similar to how a person perceives an animal, from retinal imaging through the determination that it is a horse at the end. It is challenging to articulate the message during this time since it is gradually abstracted across the neurological system at several sensory levels. However, it is important to define the message form on each hidden floor and specify its appropriate relationship with known quantities in order to train the deep Internet hierarchically [10, 11]. According to the study, the corresponding data tables are established to study and analyze them, such as Tables 1 and 2.

After continuous expansion and improvement, deep knowledge has turned into one of the most important technologies in the domain of man-made intelligence and has outstanding and excellent performance in many applied domains. An in-depth study discussed on how to automatically learn and represent the potential distribution characteristics of model data with multifloor build, which reduces the requirements for the number and labeling of sample data and automatically extracts the characteristic of various levels needed for classification across unguided training process, which has many qualities different from the existing machine knowledge techniques.

RETRACTED

### 3.2. Analysis and Study of Deep Knowledge Algorithm

Deep knowledge is a new domain of machine knowledge study. Based on neural Internet, a model simulating the analysis and knowledge of human brain is established, and the target is identified by imitating the mechanism of human brain. As the basic floor of the Internet, RBM is used to train the Internet floor by floor from bottom to top, until the required output is generated at the top floor. The training algorithm of each floor is the same: the lowest floor takes known data as input and generates data as output; each upper floor takes the output of the lower floor as input and generates data as the output of the upper floor. For example, the input can be various handwritten digital images, while the output is 0~9. The input and output dimensions of each floor, as well as the number of floors in the deep Internet, can be specified by themselves as required, without special constraints. This discovery undoubtedly adds insult to injury to the expansion of BP neural Internet, and the study of man-made neural Internet has once again come to a standstill. In this process, machine knowledge methods based on statistical ideas have gradually gained mainstream support in the industry. Decision tree, SVM, random forest, and other algorithms have been born, which have achieved good results in data classification and regression and have turned into the mainstream algorithms of machine knowledge. Deep knowledge was first applied in the domain of image recognition and achieved great success in image classification, face recognition, general object detection, image segmentation, optical character recognition, and other domains. In recent years, deep knowledge technology has been widely introduced into the domain of man-made intelligence. Almost all new intelligent voice assistants are based on deep knowledge architecture, such as Cortana of Microsoft, Xiaodi of Baidu, Iflytek, Xiaoai of Xiaomi, and Siri of Apple. At present, it has been used in commercial application, including image admit and detection, and well-known driverless cars such as Google, Tesla, and Baidu. The Institute of Botany, Chinese Academy of Sciences, cooperated with Lulang Software to identify thousands of flowers with high accuracy. Taobao's application integrates taking photos to identify goods and provides relevant links to purchase goods [12, 13]. In the study, the corresponding algorithm formula is established according to its RBM, as shown in

(1) $$\begin{array}{c} E\left(v,h\right)=-\underset{i=1}{\sum }\overset{m}{\underset{j=1}{\sum }}W_{ij}v_{i}h_{j}-\overset{n}{\underset{i=1}{\sum }}v_{i}b_{i}. \end{array}$$

Due to the fact that the conditional probability value of hidden units only depends on the distribution of explicit units, it is possible to calculate the conditional probability of hidden units using

(2) $$\begin{array}{c} p\left(h_{j}\left|v\right.\right)=\sigma \left(\overset{n}{\underset{i=1}{\sum }}w_{ij}v_{i}+c_{i}\right). \end{array}$$

Similarly, the conditional probability of explicit unit can be easily obtained as shown in

(3) $$\begin{array}{c} p\left(v_{j}\left|h\right.\right)=\sigma \left(\overset{m}{\underset{j=1}{\sum }}w_{ij}h_{i}+b_{i}\right). \end{array}$$

In contrast, the diffusion technique significantly improves the process of acquiring model rebuild values through widespread Gibbs acceptance. Significantly increase the algorithm's effectiveness as seen in

(4) $$\begin{array}{c} {Vw}_{ij}=\delta \left(<v_{i}h_{j}>-<v_{i}h_{j}{>}_{\text{recon}}\right). \end{array}$$

The performance of weak classifiers can be compared in order to determine which one performs the best, although it is challenging for weak classifiers in general to produce the desired outcomes, as indicated by

(5) $$\begin{array}{c} H_{t}\left(x_{i}\right)=1\overset{n}{\underset{j=1}{\sum }}hj\left(x_{i}\right)\geq \varphi . \end{array}$$

The feature extraction of CNN is realized by alternating convolution floor and pool floor, and its idea is to imitate human retinal sensory nerve as shown in

(6) $$\begin{array}{c} C_{i}=\left(\text{sigmoid}\left(w_{i}⊗x+b_{i}\right)\right), \end{array}$$

where *x* is the original input image, ⊗ represents convolution operation, and *i* represents the *i*-th convolution kernel. The definition of sigmoid operation follows the convolution floor, and the definition of pool floor is shown in

(7) $$\begin{array}{c} S_{i,j}={\underset{k\in \Omega_{i,j}}{\text{Max}}}^{\left\{C\left(K\right)\right\}}. \end{array}$$

Select six feature convolution kernels for the input image in floor *C*, and the calculation method of the convolved feature map-like convolution kernels is shown in

(8) $$\begin{array}{c} {\text{Ouput}}_{h}=\frac{\left(\text{orginal siz}{\text{e}}_{h}-\text{kernel siz}{\text{e}}_{h}\right)}{\text{stride}}+1. \end{array}$$

In the feature image, the pixel value *P*_*i*_ of the convolution result picture can be obtained by convolving the feature image, as shown in

(9) $$\begin{array}{c} P=WX, \end{array}$$

where *X* is the input characteristic picture and *W* is the parameter to be learned. The output characteristic picture is shown in

(10) $$\begin{array}{c} \text{Out}=f\left(p+b\right). \end{array}$$

Deep knowledge application in the field of vision and images is currently gaining popularity quickly, and its primary application scenarios include face admission, face tracking, object scene admit, and others. For instance, many smart phones currently available have a face unlocking feature. A quick and accurate input procedure is all that is required to unlock a mobile phone using facial recognition. The image admit technology, which is based on in-depth information, will continue to advance with the advancement of science and technology, and its accuracy will get closer and closer to that of humans. Deep knowledge has become increasingly important to our daily lives and production as a result of deep knowledge technology's constant advancement and growth in its application sectors.

RETRACTED

## 4. Study on the Build of New Socialistic Village

### 4.1. Analysis of New Socialistic Village Build

A four-in-one integrated concept of economy, politics, culture, and social structure is the new socialistic village. With just 20 words, the “Proposal” of the 11th Five-Year Plan sketches a stunning picture of a brand-new village: “production expand, affluent life, civilised rural style, clean village, and democratic management.” The financial fund for supporting agriculture is the direct mechanism of national finance distribution to agriculture and rural areas, reflecting the relationship between distribution between workers, peasants, and urban and rural areas. The distribution of financial spending for supporting agriculture does not prioritize economic gains, in contrast to bank loan funds. All agricultural public investment initiatives need assistance from state financial funds, even if they have mixed social and economic outcomes. The central government believes that creating a new socialist village is a crucial strategic job for resolving the “three rural issues,” realizing the objective of creating a moderately wealthy society and creating a harmonious socialist society. Its realistic foundation is growing and divided between urban and rural areas as well as the challenges faced by the sizable rural population in fairly sharing the benefits of modernization. In traditional Chinese nations, the state's coercive rule and rural self-integration are the key pillars of governance. The imperial power-bureaucracy system based on cities ruled the vast territory and large population across administrative cities scattered in different places. In order to maintain the existence and operation of the ruling machine, taxes and military service must be levied on the population living in the village. Paying taxes and military service is a natural obligation of the rural population as “subjects.” The integration of country and village is mainly an administrative integration that is not restricted by the object of integration. Enrich people's lives. Farmers' overall income is increasing, their living standards are increasing year by year, and their consumption build and living conditions are improving. At the same time, the communication between urban and rural areas is accelerating, and the influence of mass media is constantly updating farmers' ideas. The awareness of market economy, time efficiency, and reform and opening up are increasingly accepted by farmers. Message, science, culture, technology, and knowledge have turned into the common pursuit of farmers, and rural communities are transforming from a closed traditional life to an open modern life. The changes and expansion of rural communities provide the basic conditions for the establishment of a knowledge community and the build of a new socialistic village. The state has blocked the integration of urban and rural areas through a number of administrative measures and moved toward the dual social build on the basis of the dual economic build between urban and rural areas in order to ensure the priority of cities and facilitate the absorption of resources from rural areas. Three pillars make up the majority of this structure. The first is the world's tightest system for registering households and attaching land. The household registration system is strongly tied to the means of production and subsistence, social security, and social welfare in addition to being used to register the population. It is challenging for individuals to jump out of the “farm gate” in order to keep the populace securely fixed on the land. The second is a tax structure for agriculture that is based on that sector of the economy. It must pay taxes as long as it is a part of the agricultural population. Farmers' obligations have been enhanced in particular by the people's commune system [14, 15].

RETRACTED

In the study, the corresponding data charts are established as shown in Figures 3–5.

Figure 5 shows that under the background of deep knowledge, it has a certain impact on the new rural build, and its impact is as high as 54.53%. Since the implementation of the proactive fiscal policy, national debt investment has produced enormous economic, social, and ecological benefits in alleviating the serious shortage of agricultural investment in China, improving agricultural production conditions and promoting the expansion of farming and rural economy. However, it should be emphasized that at the moment, national debt funds are the primary source of support for agricultural investment and that their share of the central agricultural infrabuild investment is very substantial compared to that of the infrabuild investment in the normal budget. China's economy and society have rapidly advanced since the reform and opening up, and both urban and rural areas have undergone significant transformation. In contrast to the changes in the appearance of the city, numerous modern cities have been constructed in a variety of locations, which may be described as an affluent scene with high-rise structures, hectic traffic, and packed people. Compared to urban areas, rural areas have undergone significantly fewer changes. There are still a lot of old buildings in the central and western regions, as well as a lot of damaged houses and clay houses in certain underdeveloped areas, despite the fact that there are many modern houses in developed coastal areas and suburbs of several large and medium-sized towns. Single actions were the primary strategies used in the past to encourage rural expansion and transformation. Because there was little overall coordination, these actions were frequently implemented by various departments, which had a poor overall impact. In the construction of new rural areas, social initiatives as well as overall economic expansion are continually advanced. Farmer income is also increased, and not only material but also political, spiritual, and socially harmonious civilizations are built. The scientific idea of expansion is centered on individuals. Meeting people's many needs and fostering their overall expansion are the ultimate goals, regardless of whether the focus is on the economics, social initiatives, or infrastructure development. People are educated and cultivated by their surroundings. The poor economic and social conditions in rural regions, which are unable to support the diverse needs of people's all-around expansion, are mostly to blame for the low quality of China's rural population and labour force. Promoting the construction of new villages involves enhancing the economic and social climate in rural areas and creating favourable external conditions for the expansion of people in all spheres [16, 17].

### 4.2. Study on Evaluation Index of New Socialistic Village Build

The index system is an intuitive description of the general situation of the build of a new socialistic village. It concretes the abstract goals, draws a blueprint for the future of the new village, and enables builders to have clear directions and goals. Secondly, it will help the local public, in accordance with the spirit of the central government, adjust measures to local conditions, give classified guidance, and steadily promote the build of new socialistic village. The evaluation system can grade the existing rural conditions according to the final evaluation score, so as to scientifically measure the progress of new rural build, accurately understand and grasp all aspects in the actual process, help coordinate all aspects in the expansion process, and provide quantitative management basis for classifying and guiding the process of new socialistic rural build around the country. Thirdly, the index system can strengthen the specific guiding role of building new village in various places. By using the evaluation index system to monitor and evaluate different areas, we can find out the weak links, existing questions, and deficiencies in the process of building a new village and make clear the key points, difficulties and efforts of practical work, so as to provide scientific basis for formulating relevant decision-making measures. From then on to the early 1980s, “new village” became a social ideal. “Upstairs and downstairs, electric lights, and telephones” seemed to be an important symbol of “new village” in farmers' minds. In the early 1980s, the concept of “moderately prosperous society” was proposed, in which building a new socialistic village is one of the important contents of a moderately prosperous society. At present, the new socialistic village proposed by the CPC Central Committee is an important decision based on the basic judgment that “at present, the expand stage of ‘promote farming by industry and bringing the city to the village' has been reached, and the key and difficult point of building a moderately prosperous society in an Comprehensive is that the most arduous task in the process of building a moderately prosperous society in rural areas is to change the situation that rural economic and social expand is obviously lagging behind” [18, 19]. In the study, the corresponding data graphs are established to study and analyze them, as shown in Figures 6 and 7.

RETRACTED

From Figure 7, it can be seen that there are many factors affecting the new rural build and its indicators, and the impact is as high as 54.64%. The expansion of modern society has given the village a broader connotation, reflecting the synthesis of various social relations and spatial environment based on farming, villages, and environment, which are constantly extending and developing, including production and lifestyle, system, and ideology, and the typical form of spatial build. The new socialistic village refers to the comprehensive reflection of these domains in a specific period under socialistic conditions. Building a new socialistic village is a big systematic project involving all aspects of rural economic and social expand. From the perspective of system theory, the system has a clear boundary. To study its main influencing factors and system build, it is necessary to study the main factors affecting the build of new socialistic village from the perspective of outside the system, that is, the system environment. Secondly, it studies the main elements of the new socialistic village from the perspective of the internal build of the system. Third, it studies the main components and system build of building a new socialistic village from the perspective of comprehensive integration outside and inside the system [20].

## 5. Conclusions

Promoting the construction of a new socialist community is very important and contains a lot of information. It is a lengthy and difficult historical task that requires unceasing efforts from numerous angles. In order to be solid and steady as we encourage the construction of a new village, we must pay attention to and understand the practical operating issues. It is impossible to fully implement or even address all issues related to “farming, rural areas, and farmers” at once, let alone stimulate the construction of a new village. Different emphases should be established in accordance with the requirements of various places, as well as perhaps various stages and years. Follow the overall strategy, bring needs and opportunities together, and begin with the issues that farmers most urgently require, directly benefit from, mature practices, and are most likely to address, so that most farmers may experience tangible benefits quickly. The key to creating a new socialistic village is to give it as many resources as possible and to unleash its inner strength notwithstanding national unification. The idea is that urban and rural communities should work together to provide rural areas with cities and provide farmland with industries. Making a new village is not intended to artificially stop the growth of cities and industries; rather, it is meant to encourage and direct the expansion of rural areas alongside those of cities and industries, from urban-rural isolation to urban-rural integration. The construction of the new socialist village here is entirely distinct from that of the nearby rural area. Deep knowledge is a vast field that focuses around the deep neural internet, an algorithm whose structure is defined by millions or even billions of factors. Numerous brand-new algorithms are proposed almost on a yearly basis. The current embedded man-made intelligence era requires lightweight man-made intelligence, keeping the performance while making the neural Internet smaller. This will help to solve the problem of how to reduce the scale and message flow of deep learning algorithms while maintaining the same or stronger prediction ability.

RETRACTED

## Figures and Tables

**Figure 1:** Convolutional neural Internet build of deep knowledge.

**Figure 2:** Cyclic neural Internet diagram of deep knowledge.

**Figure 3:** Data study map of new socialistic village.

**Figure 4:** Analysis of new rural impact study.

**Figure 5:** Study and analysis of the new socialistic rural system. Data map of the study on new socialistic village under deep knowledge.

**Figure 6:** Study on the index of new socialistic village build.

**Figure 7:** Study and analysis of the new socialistic rural system.

**Table 1:** Comparison data table of different convolutional Internets.

Type	Train	Test	Precision
LeNet-5	41.06	130	88.60
CaffeNet∗	33.90	188.74	94.82
CTFAR10	42.43	152.43	88.46
AlexNet	53.87	232.72	89.75

**Table 2:** Analysis table of similar Internet build detection and comparison ability.

Neural Internet build	Convolutional neural Internet name	Precision
A	AlexNet	89.53
	CaffeNet	95.89

B	CTFAR10	88.90
	CIFAR10∗	92.6

## Data Availability

The data used to support the findings of this study are available from the corresponding author upon request.
